# Epidemiology of *β*-Lactamase-Producing Staphylococci and Gram Negative Bacteria as Cause of Clinical Bovine Mastitis in Tunisia

**DOI:** 10.1155/2019/2165316

**Published:** 2019-08-27

**Authors:** Amira Klibi, Ahlem Jouini, Ramzi Boubaker El Andolsi, Souhir Kmiha, Cherif Ben Hamda, Kais Ghedira, Safa Hamrouni, Abdeljalil Ghram, Abderrazek Maaroufi

**Affiliations:** ^1^Laboratory of Epidemiology and Veterinary Microbiology, Group of Bacteriology and Biotechnology Development, Institut Pasteur de Tunis, BP 74, 13 Place Pasteur, Belvédère, 1002 Tunis, Tunisia; ^2^University of Tunis El Manar, 2092 Tunis, Tunisia; ^3^Laboratory of Biotechnology and Valorisation of Bio-GeoRessources, Higher Institute of Biotechnology of Sidi Thabet, BiotechPole of Sidi Thabet, University of Manouba, Ariana 2020, Tunisia; ^4^Laboratory of Bioinformatics, Biomathematics and Biostatistics, Institut Pasteur de Tunis, University of Tunis El Manar (UTM), Tunisia; ^5^Faculty of Science of Bizerte, University of Carthage, 7021 Jarzouna, Tunisia

## Abstract

The aim of this study was to determine the species distribution of* Staphylococcus,* Gram negative bacteria (GNB) and the occurrence of Methicillin Resistant Staphylococci (MRS) and Extended-Spectrum *β*-lactamase- (ESBL-) producing GNB. Bacterial culture of 300 clinical mastitis milk samples from 30 different farms across different regions of Tunisia during four seasons was realized. The obtained results showed the presence of high frequency of the tested samples with a positive growth for bacteria (64%). In addition a high recovery rate of* Staphylococci *and/or GNB in these clinical mastitis milk samples (87%) was detected. In addition, a high percentage of GNB (68.2%) compared to* Staphylococcus* species (32%) was noted. Moreover, a significant variation of the number of these bacteria according to the farm location, the seasons, and cows age was detected. The highest percentage was observed in the North of Tunisia during the winter and the spring seasons in adult cows with a dominance of GNB growth. Coagulase negative* Staphylococci* (CNS) (n=11) and GNB (n=16) species were identified.* Escherichia coli* (*E. coli*) was the most frequently found bacterium followed by* Klebsiella pneumoniae. *The dominant* Staphylococcus* isolates was* S. xylosus* followed by* S. aureus *the major pathogen isolated. Methicillin resistance was confirmed by the presence of the* mec*A gene in 3* S. aureus* and 14 CNS isolates; all of these isolates were lacking the* mec*C gene. Various species of GNB, resistant to cefotaxime, were detected (n=15). ESBLs were detected on selective medium in 10* E. coli *and 4* K. pneumoniae.* All ESBL producers strains carry the* bla*CTX-M. The presence of different resistant mastitis pathogens in dairy farms may complicate therapeutic options and contaminated animals could become zoonotic agent reservoir for human.

## 1. Introduction

Bovine mastitis is one of the most costly and complex diseases of the dairy industry worldwide. It has a negative impact on animal health and productivity and poses a potential health risk for the consumers [1]. In Tunisia, 30% of dairy cows are reformed in relation to mastitis [2, 3]. Bovine mastitis is a multifactorial disease, which develops as a result of the interaction between various factors associated with the host, the specific pathogens, the environment, the season, and the farm management [4, 5]. Numerous bacterial species have been isolated from bovine mastitis cases, but historically* Staphylococci* and* Escherichia coli*, as well as other members of the family* Enterobacteriaceae*, are the most common agents of mastitis [6–8].

Mastitis pathogens may be classified into contagious, environmental, and opportunistic germs, based on their principal mode of transmission within a herd into contagious, environmental, and opportunistic pathogens [7, 9].* S. aureus* are considered as contagious pathogens, which adapt to the environment of the mammary gland and can potentially spread from cow to cow during milking. Similarly, coliforms and CNS are considered as environmental pathogens and are opportunistic bacteria of the mammary gland that may potentially be transferred from the contaminated environment to the cow mammary gland during milking [9]. Besides, the financial implications of mastitis and their importance for public health should not be overlooked.

Beta-lactam antibiotics remain the first-line treatment in veterinary medicine [10] and their extensive use in the prevention and the treatment of mastitis represent potential implications on public health through increased risk of antibiotic residues in milk and development of multidrug resistance bacteria that could possibly be transmitted to the human consumers via milk raw and its derivative products [11].

During the last five decades, methicillin resistant* Staphylococcus aureus* (MRSA) have spread as human hospital acquired pathogens (HA-MRSA) throughout the world. More recently, community-acquired CA-MRSA and livestock-associated LA-MRSA have also emerged. MRSA isolated from livestock have been increasingly reported, and zoonotic risk of transmission to humans has already been demonstrated. Methicillin resistance in staphylococci is mainly mediated by the expression of the* mec*A gene, or its homologue* mec*C, harbored the different types of the staphylococcal cassette chromosome* mec* (SCC*mec*), located on a mobile genetic element and encodes an altered penicillin-binding protein with an extremely low affinity to *β*-lactam antibiotics [12].

On the other hand, ESBL bacteria isolates have become widespread in food-producing and companion animals worldwide, representing a rapidly evolving group of enzymes that confer resistance to most beta-lactams used in human and animals [13]. Unfortunately, recent studies have reported the increasing occurrence of highly resistant ESBL-producing* Enterobacteriaceae*, mainly* E. coli*, found in milk bovine mastitis in different countries, raising a global concern for veterinary and public health [13–15] whereas ESBL-producing* K. pneumoniae* were reported in Italy, the United Kingdom, and recently Tunisia [16–18].

Better knowledge of the distribution of the pathogens involved and the antimicrobial resistance is essential for the development of means of prevention and control as well as treatment protocols. Thus, the aims of the present study were to determine species distribution of* Staphylococcus *and GNB in clinical mastitis bovine milk from different regions in Tunisia, during various seasons and to evaluate the prevalence of methicillin resistance of* Staphylococcus* species and ESBL producers of* E. coli* from cows showing clinical mastitis.

## 2. Materials and Methods

### 2.1. Sampling

Three-hundred milk samples were collected from 300 milk samples that were aseptically collected from cows suffering from clinical mastitis. Criteria defining clinical mastitis were altered milk secretion (clots, flakes, and watery, bloody, or purulent appearance), severe local (warm and/or painful udder), and general (fever) signs of inflammation. Each sample corresponds to one individual cow, and one single infected quarter was sampled per cow before any antimicrobial treatment. Samples were obtained from 30 different farms with intensive breeding across different regions in the North (n = 198 originating from 17 different farms) and the South (n =102 originating from 13 different farms) of Tunisia, during the period from October 2013 to September 2014. The sampling season was classified as winter (December-January-February), spring (March-April-May), summer (June-July-August), and autumn (September-October-November). All cows were Tunisian breed born Holstein. The ages of the animals were determined by their dentition and confirmed by the owners as young adults (3-6 yrs), adults (7-10 yrs), and old cows (> 10 yrs) [19]. The tested farms are producing milk for the owner consumption, milk bottling, or transformation to fresh cheese. Milk was collected in sterile bottles, transported in an ice box, at 4°C to the laboratory, and immediately processed.

### 2.2. Isolation and Phenotypic Identification of Bacteria

One ml of each milk sample was suspended in 9 ml of sterile saline solution for serial dilution and then plated onto ORSAB medium (Oxacillin Resistance screening Agar Base, Oxoid) and Baird-Parker (BP) agar plates for MRSA and* Staphylococci *recovery. Plates were incubated at 37°C for 24-48h. Isolates with typical staphylococci morphology were selected (one per sample) and identified using classical biochemical methods (Gram staining, oxydase, catalase, DNase, and ability to coagulate rabbit plasma (Bio-Rad)) [20].

Similarly, serial dilutions milk samples were also seeded on MacConkey agar plates and MacConkey agar containing cefotaxime (2 *μ*g/mL) for GNB and ESBLs-producers GNB recovery. All plates were incubated at 37°C for 24 h. One to three colonies from each plate were subjected to Gram staining and identified by biochemical tests [catalase, oxydase, indole, citrate, and urease].

### 2.3. Molecular Identification of Isolated Species

Confirmation of the phenotypic identity of the different isolated species was conducted using molecular methods after DNA extraction using Instagen Matrix KIT (Biorad) for* Staphylococcus* isolates and boiling methods for GNB strains. The species-specific PCR* nuc* and* uid*A genes were used for the identification of* S. aureus* and* E. coli* isolates, respectively [20, 21]. Both strains of* E. coli *ATCC 25922 and* S. aureus* ATCC 43300 were used as positive controls. The CNS strains were identified following amplification and sequencing of* sod*A gene [22]. The identification of others GNB was realized by PCR amplification and sequencing of the 16S rRNA genes [23].

### 2.4. Identification of Methicillin Resistant* Staphylococci*

Methicillin resistance was detected by oxacillin and/or cefoxitin susceptibilities using the disk-diffusion agar method, according to CLSI, 2015 [24]. Confirmation of methicillin resistance was performed by applying conventional PCR targeting the* mec*A gene [20], and* S. aureus* ATCC 43300 being used as a control strain. All* mec*A negative CNS isolates showing oxacillin or cefoxitin resistance were tested for the presence of* mec*C gene by PCR [25].

### 2.5. Phenotypic and Molecular Detection of ESBL-Producing Isolates

GNB isolates were first screened for their phenotypic identity as ESBLs-producers on MacConkey agar containing cefotaxime (2 *μ*g/mL). These presumptive ESBL-producing isolates were further confirmed by the Double-Disk Synergy Test (DDST) with cefotaxime (CTX, 30 *μ*g) and ceftazidime (CAZ, 30 *μ*g) in the proximity of amoxicillin-clavulanic acid (AMC, 30 *μ*g).* E. coli* ATCC 25922 was used as a control strain. The characterization of CTX-M type *β*-lactamases was studied by specific PCRs only in ESBL-producing strains [21].

### 2.6. Data Analysis

All the data collected within the present study were analyzed using R software, a language and environment for statistical computing [26]. Comparison between isolation rate across seasons and Tunisian regions was carried out by means of a one-way analysis of variance (ANOVA) [27] and followed by a TukeyHSD test (Tukey Honest Significant Differences). This later is a post-hoc test based on the studentized range distribution [28]. The selection criterion for significantly isolation rate variance was a p value of 0.001 or less. Comparison between percentage was performed by means of a Chi-square statistic (P < 0.01) [29]. A statistical method of assessing the significance of a difference is when the data from two or more samples is represented by a discrete number.

## 3. Results

### 3.1. Prevalence of Mastitis Pathogens

Bacterial isolates were collected, during four seasons, from 300 suspected cow milk samples with clinical mastitis, living in 30 different regions in the North and the South of Tunisia.  Table 1 shows a high proportion of positive culture of mastitis milk samples (64%). However, the percentage of negative culture samples was 36%. In addition, 87% of the tested samples showed a positive growth for* Staphylococci* and/or GNB. A total of 261 isolates was recovered with 32%* Staphylococci *(1 isolate per sample) and 68.2% GNB (1-3 isolates per sample). It is important to note that fifty five samples were polycmicrobial and contained more than one bacterial specie. Information about a sampling is shown in Table 1.

### 3.2. Relationships between Season, Region, and Mastitis Pathogens

In our study, associations between the regions, the seasons, and mastitis pathogens detected were identified through statistical-based analysis. Clinical mastitis was significantly more reported in the North compared to the South (P=0.005), with an isolation rate of 42.4% and 31%, respectively. As well, the isolation rate of positives samples with* Staphylococcus* and /or GNB recovery is higher in the North (P=2.2e-16) in comparison with the South, respectively, 79.3% and 20.7%. Significant variance between the positive culture of pathogenic bacteria across seasons was also found (P= 9.44e-06). In fact, bacteria culture was more common in the spring and in the winter rather than other seasons (Figure 1). Also during this latter, the isolation rate of environmental pathogens involved in bovine mastitis is significantly higher than that of staphylococci (P < 0.001).

### 3.3. Relationships between Age and Mastitis Bovine

Data analysis revealed a significantly higher prevalence of mastitis in adult cows (n=240; 80%) rather than in old (n=40; 13.33%) and young cows (n=20; 0.66%) with a Chi-squared p-value (P) = 2.2e-16.

### 3.4. Distribution of* Staphylococcus* Species

The numbers and the proportions of isolates of different staphylococci species are shown in Table 2. Eighty-three* Staphylococcus* strains were recovered (32%). Fifteen of these strains were identified as* S. aureus* (18%) and their antibiotic resistance mechanism is described previously by Klibi et al. [30]. Eleven different CNS species were identified as follows:* S. xylosus* (27),* S. warneri* (8),* S. chromogenes *(6),* S. sciuri *(5),* S. epidermidis *(5),* S. pasteuri *(5),* S. haemolyticus *(4),* S. succinus *(3),* S. equorum *(2),* S. saprophyticus *(2), and* S. cohnii *(1).

### 3.5. Prevalence of Gram Negative Bacteria Isolates

As shown in Tables 1 and 3, 178 GNB were isolate from three hundred clinical mastitis bovine milk samples tested (68.2%) and sixteen of different GNB were identified. Among these,* E. coli *(n=89) was the most isolated bacterium followed by* K. pneumonia *(n=30). The distribution of other isolated species was as follows:* Pseudomonas putida *(8),* Pseudomonas aeruginosa *(4),* Aeromonas *spp. (5),* Morganella morganii *(1),* Serratia marcescens *(10),* Stenotrophomonas maltophilia *(17),* Salmonella *spp. (4),* Pseudomonas pneumotropica *(2),* Achromobacter xylosoxidans *(1),* Pseudomonas mendocina *(2),* Pseudomonas argentinensis *(1),* Pseudomonas xanthomarina *(2),* Enterobacter cloacae *(1),* and Acinetobacter calcoaceticus *(1).

### 3.6. Phenotypic and Molecular Characterization of ESBL-Producing Strains

A total of 66 strains of GNB was resistant to cefotaxime and are as follows:* E. coli *(n=13),* K. pneumoniae *(n=15),* S. maltophilia *(n=17),* P. putida *(n=6),* P. aeruginosa *(n=4),* P. pneumotropica *(n=2),* S. marcescens *(n=1),* Aeromonas* spp. (n=1),* P. mendocina *(n=1),* P. xanthomarina *(n=1),* P. argentinensis *(n=1),* A. xanthomarina *(n=1),* E. cloacae *(n=1), and* M. morganii *(n=1). Ten* E. coli* and 4* K. pneumoniae* isolates were detected as ESBL-producing by phenotypic tests. The *β*-lactamase genes detected by PCR in all strains ESBL producers revealed the presence of CTX-M gene.

### 3.7. Methicillin Resistance in* Staphylococcus* Species

The disk-diffusion method indicated that 20 CNS (20/86) and 3* S. aureus* (3/15) isolates were methicillin resistant. The* mec*A gene was present in all MRSA isolates and in 14 of 20 MR-CNS isolates identified as* S. epidermidis *(4 isolates),* S. pasteuri *(4),* S. haemolyticus *(2),* S. sciuri *(1),* S. warneri *(1),* S. chromogenes *(1), and* S. cohnii *(1), all of them lacking the* mec*C [31] (Table 2).

## 4. Discussion

Overall, 64% of the milk samples contained either GNB, or staphylococci, or both germs. This frequency is of relevance and represents to our knowledge the first study performed on bovine mastitis in Tunisia. It is also interesting to note that mixed cultures were detected in 55% clinical mastitis samples. Only few studies have shown that the mastitis milk samples contain either GNB alone or both Gram negative and Gram positive bacteria [32, 33]. Nevertheless, the proportion of negative samples (36%) did not differ from that of other studies. According to the literature, about 14.5% to 38% of clinical mastitis milk samples were negative microbial growth [9, 34]. Our results showed that clinical mastitis was significantly more reported in the North compared to the South (P=0.005), with an isolation rate of 42.4% and 31%, respectively. In fact, climatologic factors could affect the incidence of clinical mastitis [33]. Some studies reported that the prevalence of dominant mastitis pathogens differs considerably between countries. Besides, even within the same country, such prevalence is always different among regions due to different farm management levels and climate [5].

In fact, the part of Northern Tunisia is characterized by low-lying Mediterranean massifs with access mainly to the beach, the sea, and the sun. The climate is Mediterranean with mild winters, hot dry summers and cool, and wet springs, all of which are climatic conditions affecting not only the geographical distribution of mastitis but also the variability of bacteria involved.

In our study, mastitis pathogens were most common in the spring and in the winter rather than other seasons. The prevalence of mastitis pathogens varied between studies; different studies showed that mastitis pathogens were most prevalent in spring [4, 5]. However, other reports showed that highest proportion of mastitis is during the winter [34]. Taking each pathogen into consideration, GNB (*E. coli *and* K. pneumoniae*) was more common in spring and winter seasons. During the spring and winter, the humidity and temperature are favorable for the development of coliform in the bedding. Opposite to our result, Zhang et al. [5] reported that cows were more likely to be infected by environmental pathogens (*E. coli* or* Streptococcus uberis*) in summer in Chinese dairy farms.

The present study of age-wise prevalence showed that the highest prevalence of mastitis was detected in adult cows. Similar observations were made by Mekebi el al. [19]. A high prevalence of clinical mastitis in the age group of 7-10 years may be due to decreased immunity of cows and resistance of bacteria to antibiotics that were indiscriminately used for the treatment of mastitis during previous infections.

Our investigation revealed a high diversity of different bacterial pathogens in clinical mastitis milk samples. Indeed, 87% of the tested samples showed a positive growth for Staphylococci and/or GNB. The percentage of GNB (68.2%) is revealed higher than that of* Staphylococcus* (32%). This is in accordance with the results reported by Oliveira et al. [35]. The predominance of this group seemed to be related environmental factors such as poor hygienic conditions, warm and humid weather, and the lack of farm cleanliness and sanitation [6]. In addition,* E. coli* (n=89) was the dominant Gram negative species reveled, followed by* K. pneumoniae *(n=30); this finding is in agreement with the study of Goa et al. [33]. Indeed,* E. coli* is ubiquitous, contagious, and opportunistic pathogen, the main reservoir being the mammary gland that is infected via the teat canal [6]. Consequently, these bacteria can spread from cow to cow or between quarters/ halves of the same animal during the milking process. Many reports showed that* Klebsiella *sp. was also the second most frequently isolated pathogen that may cause either individual clinical mastitis or outbreaks in dairy herds responding poorly to treatment which is likely a fatal outcome [33].

*S. marcescens*,* P. aeruginosa, *and* Enterobacter *sp. were the most common Gram negative species found aside* E. coli* and* K. pneumoniae *strains. These species were also described in varying proportions in previous studies [36]. In addition, a low percentage of other Gram negative species was characterized and which were considered as environmental mastitis pathogens but rare [36].

Concerning the prevalence of* Staphylococcus* species, we characterize a wide variety of CNS species (n=11). The species most often isolated in our survey from the milk of cows with clinical mastitis during this survey was* S. xylosus *(n=27) followed by* S. aureus *(n=15). The epidemiology of CNS mastitis is still unclear, but globally,* Staphylococci* are the most common mastitis-causing agent incriminated in cow mastitis, especially* S. aureus* which is the most common pathogenic germ found in mastitis [7, 32]. Nevertheless* S. xylosus* is an underestimated pathogenic CNS in bovine mastitis and was reported to induce a particularly strong increase in milk somatic cell count (SCC), comparable to* S. aureus* [37]. Otherwise, a considerable percentage of other CNS was identified (60.29%) such as* S. warneri*,* S. chromogenes*,* S. sciuri*,* S. epidermidis*,* S. pasteuri*,* S. haemolyticus*,* S. succinus*,* S. equorum*,* S. saprophyticus, *and* S. cohnii*. Recent findings suggested that some CNS such as* S. chromogenes* and* S. epidermidis* could be considered as contagious mastitis pathogens in dairy cows, while others like* S. haemolyticus* have been known to be an environmental reservoir inducing an elevation in somatic cell count as high as that seen during infections with the major pathogen* S. aureus* [8, 37].

*β*-Lactam antibiotics are widely used for intramammary treatment of bovine mastitis in Tunisia. Such act could contribute to the dissemination of MRSA in livestock and be considered as a zoonotic factor for human infection [38].

Our previous study has reported the presence of* mec*A gene in 3* S. aureus* isolates [30]. In addition in this study, the* mec*A gene has been detected in 14 MR-CNS isolates. It is important to note that various species of* Staphylococci *harbor the* mec*A gene (*S. sciuri *(1)*, S. warneri *(1),* S. epidermidis *(4),* S. haemolyticus *(2),* S. pasteuri *(4),* S. chromogenes *(1), and* S. cohnii *(1)). This feeding is in accordance with the report of Sawant et al. [39]. To the best of our knowledge, only few studies, released in Tunisia and Africa have reported on the occurrence of MRSA in cases of bovine mastitis [30, 40], and there is no published information regarding MR-CNS from bovine mastitis in Africa, yet, even though, previous surveys have shown that MR is relatively rare in* S. aureus *(from 1% to 4%) isolated from mastitis milk [30, 41]. Moreover, reports on MR-CNS associated with mastitis are rare but it has been demonstrated in* S. epidermidis*,* S. chromogenes, S. warneri, S. hyicus, S. simulants, S. haemolyticus *and* S. xylosus *[42, 43]. Methicillin-resistant CNS isolated from bovine mastitis is a special concern because of the risk of spreading the* mec* genes. Furthermore, emergence of resistance among CNS is a concern because resistance determinants may be transferred between staphylococcal species and present a risk for public health [44].

Additionally, 10* E. coli* and 4* K. pneumoniae *strains were ESBL-producing and harbored* bla* CTX-M gene. In Tunisia, CTX-M enzymes have been described in milk and recently in mastitis bovine milk [18, 45].

The resistance of mastitis pathogens to the extended-spectrum of cephalosporins through the production of *β*-lactamase is a serious clinical problem. However, to date, different studies have investigated the occurrence of ESBL-producing* E. coli* in dairy cows with mastitis [13, 15]. ESBL-producing* E. coli* isolates may be exchanged between humans and animals by various ways including direct contact and through food chain.

## 5. Conclusion

In conclusion, pathogen data were proven to be useful in recognizing temporal and regional effects on the distribution of specific mastitis-causing agents. Cows are more likely to be infected by environmental pathogens. Emergence of MRS and ESBL in cattle could hence complicate the treatment of bovine mastitis and present a zoonotic potential risk of human transmission. The application of good hygiene practices throughout the dairy industry and the prudent use of antimicrobial agents in diseases affecting dairy cows are important issues that should be addressed at the global level.

## Figures and Tables

**Figure 1:** Percentage of bacteria under seasons and Tunisian regions. (//): Significant difference (Chi-squared P < 0.001). (*∗*): Significant variance (Tukey HSD P < 0.001).

**Table 1:** Distribution of different isolated mastitis pathogens and their origins.

Farms	Number of milk Samples with mastitis	Period of sampling	Region Location	Number of positive milk samples with mastitis	Number of positive samples with *Staphylococcus *and /or Gram negative bacteria	Number of CNS	Number of *S. aureus*	Number of Gram negative bacteria	Coinfection of CNS and Gram negative bacteria
1	7	Autumn	North	4	5	1	1	3	1
2	11	Autumn	North	9	12	5	-	7	3
3	4	Winter	North	4	5	2	-	3	1
4	15	Winter	North	15	21	7	-	14	6
5	20	Winter	North	18	34	8	6	20	10
6	20		South	14	18	2	1	15	3
7	20		South	10	14	1	-	13	-
8	15	Spring	North	12	17	1	1	15	5
9	20		North	10	12	2	-	10	1
10	10		North	8	8	3	-	5	1
11	12		North	9	10	5	1	4	1
12	11	Spring	North	10	19	5	4	10	5
13	10		North	9	9	2	1	6	4
14	10	Spring	South	9	9	2	-	7	5
15	16		North	13	22	7	-	15	4
16	4	Summer	South	3	3	1	-	2	3
17	8		North	6	11	5	-	6	2
18	10	Summer	South	4	4	4	-	-	-
19	15		North	6	10	-	-	10	-
20	12		South	3	3	-	-	3	-
21	9		North	4	9	-	-	9	-
22	3	Summer	South	2	3	1	-	1	-
23	4		South	1	-	1	-	-	-
24	2		South	0	-	-	-	-	-
25	4		South	0	-	-	-	-	-
26	10	Autumn	North	9	3	3	-	-	-
27	5		North	0	-	-	-	-	-
28	3		South	0	-	-	-	-	-
29	6		South	0	-	-	-	-	-
30	4		South	0		-	-	-	-

Total	300			192	261	68	15	178	55

CNS= Coagulase-negative staphylococci; ESBL= Extended-spectrum beta-lactamases; *S. aureus= Staphylococcus aureus*; SARM=Methicillin resistant; *S. aureus;* MR-CNS= Methicillin resistant *Staphylococcus* coagulase negative.

**Table 2:** Distribution of *staphylococcus *species isolated from bovine mastitis milk samples.

Species isolated	Number of species of bacteria isolated	Methicillin-resistant isolates	*mec*A gene
*Staphylococcus coagulase positive*			

*S. aureus*	15	3	3 (*mec*A)

*CNS species*			

*S. xylosus*	27	2	0
*S. warneri*	8	3	1
*S. chromogenes*	6	1	1
*S. epidermidis*	5	4	4
*S. scuiri*	5	2	1
*S. pasteuri*	5	4	4
*S. haemolyticus*	4	2	2
*S. succinis*	3	0	0
*S. equorum*	2	1	0
*S. saprophyticus*	2	0	0
*S. cohnii*	1	1	1
*Total*	*83*	*23*	*17*

**Table 3:** Species of Gram negative bacteria isolated from bovine mastitis milk samples.

Bacteria species	Number	Number of CTX^R^ isolates	ESBL isolates
*E. coli*	89	13	10
*Klebsiella pneumoniae*	30	15	4
*Stenotrophomonas maltophilia*	17	17	0
*Serratia marcescens*	10	1	0
*Pseudomonas putida*	8	6	0
*Aeromonas *sp.	5	1	0
*Pseudomonas aeruginosa*	4	4	0
*Salmonella *sp.	4	0	0
*Pseudomonas mendocina*	2	1	0
*Pseudomonas xanthomarina*	2	1	0
*Pasteurella pneumotropica*	2	2	0
*Pseudomonas argentinensis*	1	1	0
*Acinetobacter calcoaceticus*	1	1	0
*Achrombacter xylosoxidans*	1	1	0
*Enterobacter *sp.	1	1	0
*Morganella Marganii*	1	1	0
*Total*	*178*	*66*	*14*

ESBL= Extended-spectrum beta-lactamases; CTX^R^= Cefotaxim resistant.

## Data Availability

The data used to support the findings of this study are available from the corresponding author upon request.
